The article "The Innovation of College Students' Ideological and Political Education under the Intelligent Environment of Internet of Things" was retracted in 2023. Reasons: unreliable results or conclusions; concerns about the data; concerns about the peer review; concerns about the citations.

# The Innovation of College Students' Ideological and Political Education under the Intelligent Environment of Internet of Things

**DOI:** 10.1155/2022/6420262

**Published:** 2022-06-30

**Authors:** Xia Wang

**Affiliations:** College of Maxism, Qingdao HuangHai University, Qingdao, Shandong 266427, China

## Abstract

With the development of the times and the continuous improvement of the requirements for college students' political literacy and identity, the informatization reform and educational innovation of college students' ideological and political education have become the focus and difficulty of teaching reform. The ideological and political education in most domestic colleges and universities still focuses on the elaboration of theoretical knowledge, ignoring the importance of social practice. Therefore, this paper puts forward the research on the innovation of college students' ideological and political education in the intelligent environment of the Internet of things, constructs the college ideological and political education training cloud system through the Internet of Things technology and AR technology, and promotes the realization of the purpose of college students' participation in social practice. The experimental results show that the college ideological and political education training cloud system based on AR and Internet of Things technology can improve the interaction and participation of ideological and political courses, stimulate students' interest and enthusiasm, deepen students' understanding of the content of ideological and political education, and better understand the importance of ideological and political education. At the same time, the system is also the exploration and practice of teaching innovation of ideological and political education in the intelligent environment of Internet of Things. It is a new attempt of ideological and political education reform in colleges and universities.

## 1. Introduction

Ideological and political education is not only the core embodiment of political socialization, but also the bearer of the transmission of values and beliefs of the political system [1]. The attitude of social members toward the political system will be affected by ideological and political education to a great extent. Since entering the new era, college students can be exposed to different values and information transmission in the Internet environment, and their value judgment is easy to be affected [2]. With the continuous development and evolution of the domestic and international situation, college students need to further strengthen their political literacy and identity, so as to meet the challenges of higher requirements. In recent years, colleges and universities have been strengthening and improving students' ideological and political education [3]. With the development of the times, they have continuously improved educational contents and means and achieved certain results [4]. However, there are still some problems in the ideological and political education in domestic colleges and universities, such as boring, obscure, abstract, and difficult to understand, which makes it difficult for college students to have personal experience [5]. At the same time, in terms of educational means, it still focuses on theoretical teaching, ignoring the importance of practical teaching, and the single teaching means and methods are also difficult to meet the needs of college students [6]. Therefore, how to innovate ideological and political education in colleges and universities under the background of the new era has become the research hotspot and focus of college education [7]. The theoretical content of ideological and political education in colleges and universities should not only focus on the interpretation of theoretical knowledge and theoretical system in ideological and political teaching materials [8] but also should fully tap the ideological and political education resources contained in various courses, connect ideological and political education with general courses and professional courses in colleges and universities, and explain the ideological and political theoretical knowledge from different angles. In addition, education needs the unity of knowledge and practice [9]. The ideological and political education of college students should carry out social practice on the basis of learning theoretical knowledge and expand the ways of ideological and political education in different ways.

The article "The Innovation of College Students' Ideological and Political Education under the Intelligent Environment of Internet of Things" was retracted in 2023. Reasons: unreliable results or conclusions; concerns about the data; concerns about the peer review; concerns about the citations.

This paper puts forward the research on the innovation of college students' ideological and political education in the intelligent environment of Internet of things and constructs the practical training cloud system of college ideological and political education combined with AR technology and Internet of things technology. This paper is mainly divided into three parts. The first part expounds the communication means of ideological and political education; The second part is the construction of college ideological and political education and training cloud system based on AR and Internet of things technology. The third part is the application effect analysis of college ideological and political education and training cloud system based on AR and Internet of things technology. The research provides technical support for the improvement of the ideological and political education system in colleges and universities and widens the realization ways of ideological and political education in colleges and universities.

## 2. Communication Means of Ideological and Political Education

Ideological and political education plays an important role in any country. Different countries realize the purpose of ideological and political education through different means of communication based on their own cultural background and combined with practical needs [10]. Most foreign ideological and political education combines civic education, moral and legal education, religious education, and history education [11]. For example, the United States pays more attention to creating a moral and cultural atmosphere in the dissemination of ideological and political education, that is, cultivating students' virtues and consolidating the core values of the school through communication means such as teaching building banners, classroom decoration, school newspapers and magazines, blackboard newspaper, and so on [12]. At the same time, the United States continues to explore how to achieve the purpose and effect of civic education through the Internet platform. The United Kingdom focuses on the combination of mass media and academic circles to realize the civic education of teenagers, that is, teenagers acquire civic knowledge through the Internet, civic moral education, television, radio columns, and other channels [13]. Compared with Britain and the United States, Russia's means of communication in patriotism education are relatively more diversified, mainly divided into two parts: the innovative use of traditional media and the use of Internet. In the innovative use of traditional media, Russia will specially set up patriotic TV channels, film patriotic themes, and publish educational books on relevant themes [14]. At the same time, Russia will also set up websites and social platforms for teenagers through the Internet, and design and develop games with patriotism as the theme. Japanese colleges and universities have divided the content of ideological and political education into five categories, namely patriotism education, outlook on life education, personality and group education, international interaction, and labor education [15]. While conducting some theoretical education of ideological and political education through mass communication, they also pay attention to the application of practical methods of ideological and political education, such as taking students on field trips to local areas [16]. To sum up, although foreign universities have different communication contents of ideological and political education, there are still many common points in their communication means and methods, which can be continuously improved and innovated with the development of the times [17]. It not only integrates the needs of local characteristic culture and contemporary culture into the traditional mass communication mode to create a good ideological and political education atmosphere for colleges and universities but also constantly discusses and learns to use modern network communication mode to strengthen the teaching effect of ideological and political education.

The article "The Innovation of College Students' Ideological and Political Education under the Intelligent Environment of Internet of Things" was retracted in 2023. Reasons: unreliable results or conclusions; concerns about the data; concerns about the peer review; concerns about the citations.

In China, ideological and political education is one of the compulsory courses for college students, and ideological and political education also realizes the effect of communication education in colleges and universities through two ways: intraorganizational communication and interpersonal communication. As a public medium, campus media in the organizational communication channel includes traditional media means, such as campus radio, television, and periodicals, as well as new media forms, such as campus website, mobile app, and QQ group [18], which makes the communication of ideological and political education in colleges and universities have the characteristics of high exclusivity and credibility. With the development of Internet and social media, colleges and universities explore the communication value of social network as a new means of ideological and political education from the needs of college students' emotion and will. Ideological and political educators have strengthened the interaction and communication with students through wechat, microblog, live broadcast, and other social media, and have a more comprehensive and multiangle understanding of students' state of mind [19]. At the same time, some scholars of ideological and political education pointed out that digital media means have stronger information media interaction than traditional media means and can optimize information communication tools, but at the same time, negative information is also easy to appear in the massive information and content. This requires the active use of digital media means for ideological and political education communication, while improving and perfecting the mechanism of digital communication. With the continuous development of digital media and new media means, domestic ideological and political educators should actively try to change the ideas and ways of ideological and political education, explore new communication means of ideological and political education and improve the informatization degree of ideological and political education [20].

## 3. Construction of College Ideological and Political Education Training Cloud System based on AR and Internet of Things Technology

The practical training cloud system of Ideological and political education in colleges and universities based on AR and Internet technology mainly includes background management function, NFC recording function, on-site AR function, and on-site team training function. On the basis of meeting the requirements of the intelligent environment of the Internet of things and the integration of ideological and political education, it greatly reduces the cost of organizing and carrying out social practice of ideological and political education in colleges and universities.

The article "The Innovation of College Students' Ideological and Political Education under the Intelligent Environment of Internet of Things" was retracted in 2023. Reasons: unreliable results or conclusions; concerns about the data; concerns about the peer review; concerns about the citations.

This system consists of the information release system V1.0 of ideological and political course education and teaching resource database 0 software and a remote group construction device for ideological and political education based on ar-nfc. It is the crystallization of NFC technology, AR technology, Internet of things technology, mobile communication technology, cloud database technology, and other advanced technologies. The system can effectively solve the problems encountered in the current ideological and political education and teaching in colleges and universities, which is worthy of reference and popularization and application. As shown in Figure 1, it is the overall framework of college ideological and political education and training cloud system based on AR and Internet technology. As can be seen from the figure, the system group should be divided into two parts. The upper part is ar NFC type ideological and political education remote group construction equipment, and the lower part is an external cooperation system, which can be connected with multiple remote group construction equipment.

This paper mainly expounds the Internet of things development and access point technology based on near-field communication induction, that is, NFC induction, and virtual reality based on AR scene in the college ideological and political education training cloud system based on AR and Internet technology.

### 3.1. Internet of Things Development and Access Point Technology based on NFC

In addition, NFC technology provides the possibility for mobile phones to realize the work of Internet of things access system under the condition of low-power consumption, and its performance is better than infrared technology and Bluetooth technology. Therefore, the Internet of things development technology based on NFC is also combined with android app development technology to realize the function of sensing proximity and triggering of NFC card through the development of mobile app. At the same time, three triggers can be triggered by reading the on-site NFC sensing code. As shown in Figure 2, it is the flow chart of Internet of things technology based on NFC sensing.

The article "The Innovation of College Students' Ideological and Political Education under the Intelligent Environment of Internet of Things" was retracted in 2023. Reasons: unreliable results or conclusions; concerns about the data; concerns about the peer review; concerns about the citations.

College ideological and political education training cloud system access to the Internet of things needs to be realized through NFC module. From the perspective of security defense system, the security of Internet of things can also be divided into perception layer security, network layer security, and application layer security according to the architecture of Internet of things. The design of perception layer security needs to consider the limitations of computing power, communication capacity, and storage capacity of Internet of things devices. Complex security technologies cannot be directly applied to physical devices. Network layer security is used to ensure communication security, while application layer focuses on the security of various businesses and business-support platforms. At the same time, the antenna-coupling mode of NFC module can help the system obtain power supply energy from the mobile phone. RFID chip realizes data and energy interaction with mobile phones through antenna connection. The inductance of NFC antenna coil is lant, which needs to add parallel capacitance cant and serial resistance rant during equivalence. Cant represents the capacitance loss between coils and connectors, and rant represents the resistance loss. The inductance of antenna coil is calculated as shown in formula (1):

(1) $$\begin{array}{c} L\left[\text{nH}\right]=2\cdot l\left[\text{cm}\right]\cdot \left(\ln\left(\frac{l}{D}\right)-K\right)\cdot N^{1.8}, \end{array}$$

where the length of one coil of wire ring is expressed as *l*, the width of PCB wire or the diameter of coil is expressed as *D*, the number of coil turns is expressed as *N*, and *K*=1.47 if the antenna is rectangular.

Since rant cannot directly calculate the accurate value, its estimation formula is shown in formula (2):

(2) $$\begin{array}{c} \text{Rant}=5\cdot R_{\text{DC}}, \end{array}$$

where the DC resistance is expressed as *R*_DC_.

The quality factor of the antenna can reflect the correct tuning and performance index of the antenna, and its calculation formula is shown in formula (3):

(3) $$\begin{array}{c} Q=\frac{\omega_{R}\cdot L_{\text{ant}}}{R_{\text{ant}}},\\ \omega_{R}=2\pi f_{R}. \end{array}$$

In this paper, the pH sensor module based on OTFT is selected in the sensor module. In the module, MCU can only input the voltage value, so it needs resistance voltage division to transform the current signal and voltage signal. OTFT has poor performance in uniformity due to its large resistance value and low mobility. In order to better determine the resistance value, this paper selects diodes of the same material as OTFT as resistors for voltage division. As shown in formulas (4) and (5), it is the expression of drain current:

(4) $$\begin{array}{c} I_{D}=\frac{1}{2}\mu C_{G}\frac{W}{L}{\left(V_{GS}-V_{\text{th}}\right)}^{2}, \end{array}$$

(5) $$\begin{array}{c} I_{D}=\mu C_{G}\frac{W}{L}\left(V_{GS}-V_{\text{th}}\right)V_{DS}, \end{array}$$

where the drain current is expressed as *I*_*D*_, the mobility of OTFT is expressed as *μ*, the capacitance per unit area of gate insulating layer is expressed as *C*_*G*_, the channel width is expressed as *W*, the channel length is expressed as *L*, the threshold voltage is expressed as *V*_th_, and the gate source voltage is expressed as *V*_*GS*_ and *V*_*GS*_=*V*_*in*_ − *V*_*dd*_, where *V*_*in*_ is the input voltage and *V*_*dd*_ is the supply voltage.

The article "The Innovation of College Students' Ideological and Political Education under the Intelligent Environment of Internet of Things" was retracted in 2023. Reasons: unreliable results or conclusions; concerns about the data; concerns about the peer review; concerns about the citations.

The circuit conduction current of pH sensor-voltage output is related to the ratio of driving OTFT aspect ratio and load aspect ratio. If the ratio is expressed as *N*, the relationship between voltage and input voltage under different *N* values is shown in Figure 3:

It can be seen from the figure that due to the poor uniformity of OTFT, there are obvious differences in the performance of different voltage output circuits based on OTFT. Therefore, it is necessary to calibrate to make the voltage output circuit have good consistency in the actual measurement. In the actual measurement process, the function of the reference voltage with respect to the output voltage can be obtained, that is, *V*_ref_=*f*(*V*_out_), where *V*_ref_ represents the reference voltage and *V*_out_ represents the output voltage. When the standard buffer solution of *PH*=4 and *PH*=10 is calibrated through the circuit, its sensitivity is shown in formula (6):

(6) $$\begin{array}{c} \text{sensitivity}=\frac{V_{\text{ref},10}-V_{\text{ref},4}}{10-4}. \end{array}$$

The calculation formula of pH value is shown in formula (7):

(7) $$\begin{array}{c} \text{PH}=\frac{V_{\text{ref},7}-f\left(V_{\text{out}}\right)}{\text{sensitivity}}+7. \end{array}$$

When the Android mobile phone uses the pH sensor label for the first time, it needs to be calibrated, that is, the mobile phone will receive 25 pairs of data sent by the wireless access module and use these data to build the functional relationship between the output voltage and the input voltage. Therefore, this paper selects the Boltzmann model for fitting, and its expression is shown in formula (8):

(8) $$\begin{array}{c} y=\frac{A_{1}-A_{2}}{1+e^{\left(x-x_{0}\right)/\text{d}x}}+A_{2}, \end{array}$$

where *A*_1_, *A*_2_, *x*_0_, d*x* is the parameter.

### 3.2. Virtual Reality Technology based on AR Scene

Augmented reality technology, AR technology, is a derivative technology of virtual reality technology, which involves many technologies such as digital image processing, computer vision, and so on. AR technology superimposes the generated virtual information and the real scene image through the calculation of the influence position and angle of the camera, enhances the user's visual perception of the real world through the rendering of the virtual reality fusion effect, and presents the scene of parallel interaction between the virtual world and the real world on the mobile phone screen. The cloud system of ideological and political education training in colleges and universities imports the photos and other materials of real scenes into the cloud database through the background program through AR technology, and generates the corresponding ar induction code. Each ar induction code corresponds to a scene, and each scene contains multiple materials, and each material corresponds to problems in single or multiple cloud databases. In this way, the function of random extraction can be realized at the same time.

The article "The Innovation of College Students' Ideological and Political Education under the Intelligent Environment of Internet of Things" was retracted in 2023. Reasons: unreliable results or conclusions; concerns about the data; concerns about the peer review; concerns about the citations.

The key to the perfect and seamless integration of real scene and virtual object through AR technology is that when the relative position of camera and object in real scene changes, the corresponding registration position of virtual object will also change. The geometric model of camera imaging determines the corresponding relationship between them. In computer vision, the camera imaging process involves three very important coordinate systems, namely image coordinate system, camera coordinate system, and world coordinate system. The representation of image coordinate system is generally expressed in pixel units and physical units. Let the rectangular coordinate system be *O*_0_*uv*, a coordinate in the pixel coordinate system be represented as (*u*, *v*), the corresponding physical position coordinate of the pixel in the image be represented as (*x*, *y*), and the origin *O*_1_ of the physical coordinate system be the intersection of the camera optical axis and the plane, which is represented as (*u*_0_, *v*_0_) in the pixel coordinate system. The size of the unit pixel scale of a pixel in the image in the horizontal axis and vertical axis directions is expressed as *k*, *l* respectively, then the relationship between the pixel coordinates and physical coordinates is shown in formulas (9) and (10):

(9) $$\begin{array}{c} u=\frac{x}{k}+u_{0}, \end{array}$$

(10) $$\begin{array}{c} v=\frac{y}{l}+v_{0}. \end{array}$$

The matrix and its inverse representation are shown in formulas (11) and (12):

(11) $$\begin{array}{c} \left[\begin{array}{c} u\\ v\\ 1 \end{array}\right]=\left[\begin{array}{ccc} \frac{1}{k} & 0 & u_{0}\\ 0 & \frac{1}{l} & v_{0}\\ 0 & 0 & 1 \end{array}\right]\left[\begin{array}{c} x\\ y\\ 1 \end{array}\right], \end{array}$$

(12) $$\begin{array}{c} \left[\begin{array}{c} x\\ y\\ 1 \end{array}\right]=\left[\begin{array}{ccc} k & 0 & -u_{0}k\\ 0 & l & -v_{0}l\\ 0 & 0 & 1 \end{array}\right]\left[\begin{array}{c} u\\ v\\ 1 \end{array}\right]. \end{array}$$

The homogeneous coordinates of camera coordinate system and world coordinate system are (*X*_*W*_, *Y*_*W*_, *Z*_*W*_, 1), (*X*_*C*_, *Y*_*C*_, *Z*_*C*_, 1), and the transformation relationship between them is shown in formula (13):

(13) $$\begin{array}{c} \left[\begin{array}{c} X_{C}\\ Y_{C}\\ Z_{C}\\ 1 \end{array}\right]=\left[\begin{array}{cc} R_{3\times 3} & t_{3\times 1}\\ 0^{T} & 1 \end{array}\right]\left[\begin{array}{c} X_{W}\\ Y_{W}\\ Z_{W}\\ 1 \end{array}\right], \end{array}$$

where *R*_3×3_=(*r*_*x*_, *r*_*y*_, *r*_*z*_) represents the orthogonal unit rotation matrix and *r*_*x*_, *r*_*y*_, *r*_*z*_ represents the rotation component on the three coordinate axes. $t_{3\times 1}=\left[\begin{array}{c} t_{x}\\ t_{y}\\ t_{z} \end{array}\right]$ is the translation vector, 0=(0,0,0)^*T*^.

The article "The Innovation of College Students' Ideological and Political Education under the Intelligent Environment of Internet of Things" was retracted in 2023. Reasons: unreliable results or conclusions; concerns about the data; concerns about the peer review; concerns about the citations.

The perspective projection relationship of pinhole camera model is shown in formulas (14) and (15):

(14) $$\begin{array}{c} x=\frac{fX_{C}}{Z_{C}}, \end{array}$$

(15) $$\begin{array}{c} y=\frac{fY_{C}}{Z_{C}}. \end{array}$$

In the formula, the image physical coordinate of a point in space on the two-dimensional image is expressed as (*x*, *y*), and the coordinate under the camera coordinate system is expressed as (*X*_*C*_, *Y*_*C*_, *Z*_*C*_). The relationship between the point's world coordinate (*X*_*W*_, *Y*_*W*_, *Z*_*W*_) and its projected image pixel coordinate on the two-dimensional image plane is shown in formula (16):

(16) $$\begin{array}{c} Z_{C}\left[\begin{array}{c} u\\ v\\ 1 \end{array}\right]=\left[\begin{array}{ccc} \frac{1}{k} & 0 & u_{0}\\ 0 & \frac{1}{l} & v_{0}\\ 0 & 0 & 1 \end{array}\right]\left[\begin{array}{cccc} f & 0 & 0 & 0\\ 0 & f & 0 & 0\\ 0 & 0 & 1 & 0 \end{array}\right]\left[\begin{array}{cc} R_{3\times 3} & t_{3\times 1}\\ 0^{T} & 1 \end{array}\right]\left[\begin{array}{c} X_{W}\\ Y_{W}\\ Z_{W}\\ 1 \end{array}\right]\\ =\left[\begin{array}{cccc} a_{x} & 0 & u_{0} & 0\\ 0 & a_{y} & v_{0} & 0\\ 0 & 0 & 1 & 0 \end{array}\right]B\left[\begin{array}{c} X_{W}\\ Y_{W}\\ Z_{W}\\ 1 \end{array}\right]\\ =KB\left[\begin{array}{c} X_{W}\\ Y_{W}\\ Z_{W}\\ 1 \end{array}\right], \end{array}$$

where *a*_*x*_=*f*/*k*, *a*_*y*_=*f*/*l* and *K* are the internal parameter matrix of the camera, the external matrix is *B*, and *KB* is the projection matrix.

The article "The Innovation of College Students' Ideological and Political Education under the Intelligent Environment of Internet of Things" was retracted in 2023. Reasons: unreliable results or conclusions; concerns about the data; concerns about the peer review; concerns about the citations.

In order to make 3D virtual objects that can be superimposed into the real scene in real time, 3D registration is needed. The key problem is to clarify the relationship between different coordinate systems. Let the coordinate system of the virtual object be *X*_*V*_*Y*_*V*_*Z*_*V*_, and the conversion relationship between it and the world coordinate system is shown in formula (17):

(17) $$\begin{array}{c} \left(X_{W}Y_{W}Z_{W}1\right)=O\left(X_{V}Y_{V}Z_{V}1\right). \end{array}$$

Then, after the conversion between the real-world coordinate system and the camera coordinate system and the conversion between the camera coordinate system and the image coordinate system, the position of the virtual object in the two-dimensional image plane can be obtained, as shown in formula (18):

(18) $$\begin{array}{c} Z_{C}\left(uv1\right)=\text{OCP}\left(X_{V}Y_{V}Z_{V}1\right). \end{array}$$

## 4. Analysis

### 4.1. PH Measurement of Cloud System Sensor in College Training

As shown in Figure 4, the calibration curve and pH measurement value are obtained through the pattern search algorithm. The input voltage at the point with the largest derivative obtained by deriving the calibration curve is taken as the best measurement point, and the pH buffer solution to be measured is measured accordingly, and then the output voltage of the measured pH sensor label is marked on the curve. It can be seen from the output characteristic curve in the figure that when the output voltage reaches *V*_out2_ and the corresponding input voltage is *V*_ref2_, the implementation of the algorithm is the solution process of the inverse function of the Boltzmann function of the output and input voltage, and then calculate the sensitivity of the pH tag. After the pH tag is put into the pH solution to be tested, repeat the process to obtain the corresponding input voltage value, and finally, obtain the pH value of the buffer solution of the pH to be tested according to the pH calculation formula.

### 4.2. Application Results of College Ideological and Political Education Training Cloud System based on AR and Internet of Things Technology

In order to better understand the application effect of college ideological and political education training cloud system based on AR and Internet of things technology, this paper conducted an ideological and political education training experiment for a college student. The number of participants in the experiment is 185. According to the relevant survey results, 47 students like ideological and political courses in colleges and universities, 30 students do not like ideological and political courses in colleges and universities, and the other students maintain a neutral attitude toward ideological and political courses. It can be seen that although colleges and universities take ideological and political education as a compulsory course, most college students do not pay attention to ideological and political education, and their interest and liking for the course content are not high as a whole.  Figure 5 shows the survey results of the reasons why college students like and dislike ideological and political courses.

The article "The Innovation of College Students' Ideological and Political Education under the Intelligent Environment of Internet of Things" was retracted in 2023. Reasons: unreliable results or conclusions; concerns about the data; concerns about the peer review; concerns about the citations.

As shown in Figure 6, it is the evaluation results of students on the current ideological and political courses and education in colleges and universities.

It can be seen from the data in the figure that 85.11% of the students who like ideological and political courses think the teaching methods of teachers are interesting, while 73.33% of the students who do not like ideological and political courses think the teaching contents of teachers are boring. In addition, 53.51% of the students pointed out that the current ideological and political education content and teaching methods are single, which does not meet the needs of college students. It can be seen that the teaching contents and methods of ideological and political education have a great impact on college students' liking for ideological and political courses. In addition, among the reasons why they do not like ideological and political courses, half of the students think that ideological and political education courses are divorced from the reality of life and are not helpful to their own life. This shows that the ideological and political education curriculum in colleges and universities is biased toward theoretical elaboration and ignores the importance of social practice, which makes the ideological and political education curriculum lack of interaction and participation.

As shown in Figures 7 and 8, it is the degree and reason why college students like the ideological and political course after participating in the ideological and political education training experiment.

It can be seen from the results in the figure that after participating in the ideological and political education training experiment, college students have greatly improved their liking for the ideological and political course, and the number of people who do not like the ideological and political course has also decreased significantly. It can be seen from the reasons that 70.3% of the students are interested in the teaching method of the ideological and political course, 51.89% of the students think that through this way, they can have a deeper understanding of the content of the ideological and political course, and 42.16% of the students think that such an ideological and political course can help shape their three outlooks and have a deeper understanding of the importance of ideological and political education. In addition, 64.86% of students like the interaction and participation of ideological and political courses, which improves students' enthusiasm and sense of participation.

The article "The Innovation of College Students' Ideological and Political Education under the Intelligent Environment of Internet of Things" was retracted in 2023. Reasons: unreliable results or conclusions; concerns about the data; concerns about the peer review; concerns about the citations.

To sum up, the application of college ideological and political education training cloud system based on AR and Internet of things technology improves the interaction and participation of ideological and political courses, provides college students with the opportunity to participate in the courses in person, and improves students' interest and enthusiasm in ideological and political courses. The interesting teaching method is conducive to improving students' liking for ideological and political courses, so that more students can truly understand and understand the content and importance of Ideological and political courses. At the same time, the practical training cloud system of ideological and political education in colleges and universities based on AR and Internet of things technology explores and practices the innovative education model of online and offline connection, extracurricular and in class connection.

## 5. Conclusion

This paper puts forward the research on the innovation of college students' ideological and political education in the intelligent environment of the Internet of things and constructs the ideological and political education training cloud system through the Internet of things technology and AR technology to realize the purpose of students' participation in the practical activities of ideological and political education. The experimental results show that the application of college ideological and political education and training cloud system based on AR and Internet of things technology improves the interaction and participation of ideological and political courses. It provides college students with the opportunity to personally participate in the course and improves their interest and enthusiasm in the ideological and political course. Interesting teaching method is conducive to improve students' love of ideological and political course, so that more students can truly understand and understand the content and importance of ideological and political course. At the same time, the college ideological and political education training cloud system based on AR and Internet of things technology explores and practices the innovative education mode of online and offline docking and extracurricular classroom docking. However, the curriculum of ideological and political education in colleges and universities can not only rely on AR and network technology. Ignoring the importance of social practice will make the ideological and political education curriculum lack of interaction and participation. In addition, the application of college ideological and political education training cloud system based on AR and Internet of things technology is the exploration and practice of the innovative mode of ideological and political education. In the future, we need to further compare the test results of ideological and political problems after AR experience and optimize the conclusions.

The article "The Innovation of College Students' Ideological and Political Education under the Intelligent Environment of Internet of Things" was retracted in 2023. Reasons: unreliable results or conclusions; concerns about the data; concerns about the peer review; concerns about the citations.

## Figures and Tables

**Figure 1:** Overall framework of college ideological and political education training cloud system based on AR and Internet technology.

**Figure 2:** Flow chart of Internet of things technology based on NFC sensing.

**Figure 3:** Relationship between voltage and input voltage under different values.

**Figure 4:** The calibration curve and pH measurement value are obtained by pattern search algorithm.

**Figure 5:** Investigation results of the reasons why college students like and dislike ideological and political courses.

**Figure 6:** Students' evaluation results of ideological and political courses and education in colleges and universities.

**Figure 7:** How much college students like the ideological and political course after participating in the ideological and political education training experiment.

**Figure 8:** Reasons why college students like the ideological and political course after participating in the practical training experiment of ideological and political education.

## Data Availability

The data used to support the findings of this study are available from the corresponding author upon request.
